# An Adaptive ECG Noise Removal Process Based on Empirical Mode Decomposition (EMD)

**DOI:** 10.1155/2022/3346055

**Published:** 2022-08-17

**Authors:** Ahmed. F. Hussein, Warda R. Mohammed, Mustafa Musa Jaber, Osamah Ibrahim Khalaf

**Affiliations:** ^1^Biomedical Engineering Department, College of Engineering, Al-Nahrain University, Baghdad 10072, Iraq; ^2^Department of Medical Instruments Engineering Techniques, Dijlah University College, Baghdad 10021, Iraq; ^3^Department of Medical Instruments Engineering Techniques, Al-Farahidi University, Baghdad 10021, Iraq; ^4^Al-Nahrain Nano Renewable Energy Research Center, Al-Nahrain University, Baghdad 64074, Iraq

## Abstract

The electrocardiogram (ECG) is a generally used instrument for examining cardiac disorders. For proper interpretation of cardiac illnesses, a noise-free ECG is often preferred. ECG signals, on the other hand, are suffering from numerous noises throughout gathering and programme. This article suggests an empirical mode decomposition-based adaptive ECG noise removal technique (EMD). The benefits of the proposed methods are used to dip noise in ECG signals with the least amount of distortion. For decreasing high-frequency noises, traditional EMD-based approaches either cast off the preliminary fundamental functions or use a window-based methodology. The signal quality is then improved via an adaptive process. The simulation study uses ECG data from the universal MIT-BIH database as well as the Brno University of Technology ECG Quality Database (BUT QDB). The proposed method's efficiency is measured using three typical evaluation metrics: mean square error, output SNR change, and ratio root mean square alteration at various SNR levels (signal to noise ratio). The suggested noise removal approach is compatible with other commonly used ECG noise removal techniques. A detailed examination reveals that the proposed method could be served as an effective means of noise removal ECG signals, resulting in enhanced diagnostic functions in automated medical systems.

## 1. Introduction

In the last few decades, the automated processing of physiological signals has become a hot topic. The aim of automation is to decrease the amount of time and effort, which is vital for research and construction by humans. This helps to manage a large amount of data for quick processing and decision-making, which is especially useful in intensive care facilities. Long interval biomedical data are compressed and stored in storage components in certain cases, then analysed and assessed by specialists later to identify any anomalies. Individuals with severe and numerous anomalies include simultaneous examination of multiple physiological signals. In the context of an assistive diagnosis and monitoring system, computer-based automated processes help a lot in this application [1, 2].

Electrocardiogram (ECG) is generally used for detecting cardiovascular ailments. ECG signifies the electrical actions of the cardiac system. A clinical information conveys in standard morphology of every component in the ECG rhythm. The true state of the heart can be determined by mining thorough information of every section [3, 4]. Because of the swift rise in populace and dearth of appropriate infrastructure, computer-based automated ECG analysers have emerged as a crucial means for early diagnosis of cardiac ailments, thanks to their swifter processing [5, 6]. Nonetheless, for accurate ECG signal feature extraction, noise-free and good quality signals are usually desired. In the real setting, different noises such as Gaussian noise and baseline wander noise, power line interference, and muscle artefacts corrupt the ECG wave all through its receipt and transmission [7–9]. Gaussian noise is produced when a signal is transmitted over a poor source. Muscle objects, also known as electromyograms (EMGs), are random noises that extend through the entire frequency range and are produced by multiple muscle movements. Power line noise then creates difficulties according to the main frequency of 50 or 60 Hz. Baseline wander noise is generated by the patient's respiration, which allows the reference potential point to deviate from null. The removal of such sounds is important for the correct detection of cardiac disorders dependent on signal characteristics. As a consequence, ECG signal denoising is critical and computer-based automatic ECG denoising methods are a challenging research field [10–13].

Several studies have contributed many reviews to propose the formulation of techniques for computerised ECG denoising. Such developed methods are primarily based on deep learning techniques [14, 15], deep recurrent neural networks (RNN) [16], filter banks [17], time-frequency techniques [18–20], discrete wavelet transform (DWT) filtering [21,22], empirical mode decomposition (EMD) [23–26], impulse response (FIR) filter [17, 27], nonlocal mean (NLM) filter [28], and principle component analysis (PCA) [29, 30].

Nevertheless, FIR-based filtering methods [17] can enable one to eliminate the noise frequencies which are beyond the variety of frequency of ECG signals. Furthermore, these techniques do not retain the ECG components of low frequency (P and *T* waves). Systems based on neural networks [14, 15] involve additional training stage and representative signals, hence they are not appropriate for real-time requests. In PCA methods [29, 30], the resulting numerical model is greatly complex to a small variation in the waves or even the noises. The efficiency of a NLM filter [28] is dependent on the accurate choice of structure bandwidth that can be computed from the artefacts' ST (standard deviation). In the real-world scenario, the standard deviation-based estimation of the artefacts is not feasible which results in low quality performance. DWT [21, 22] derived hard and soft thresholding-based noise removal is prevalent for nonstationary signals filtering. The filter type that employs a wavelet technique is not able to preserve the edges well. Additional technique based on EMD is pretty operative for processing the electrocardiogram signs. In this method [23], the sample signals are disintegrated into a group of oscillatory fundamentals, which are called IMF (intrinsic mode functions). The noise elements are chiefly distributed over limited low guideline IMFs. Some low-order IMFs are deleted, resulting in significant data loss in the restored ECG signals. To keep the noise elements in the QRS regions, a window is chosen in the low-order IMFs. The ADTF (adaptive dual threshold filter)-based approach [19] discards the wavelet disintegrated signal's preliminary sub-bands, resulting in substantial information loss in the higher frequency band. Furthermore, it uses a single amplitude threshold for peak correction, which is likely to fail to detect the peaks correctly in irregular ECG and time-varying QRS morphology conditions.

In this paper, an adaptive technique based on EMD to eliminate ECG noise is proposed. The proposed technique makes use of mean value for adaptive biasing to reduce IMF component (1st and 2nd) and then rebuild the original signal from the nonmodified and modified IMFs. This way ensures the noise filtering with minimum distortion. Besides, the EMD technique can be achieved by regular hardware and combining into an Internet of Thing (IoT) gadgets easily which is a benefit for automated healthcare features.

## 2. Materials and Methods

A description of the recommended approach is given in Figure 1. More details are discussed in this segment.

### 2.1. Database

For the proposed scheme of ECG denoising approach efficiency validation, datasets signals of ECG taken from MIT-BIH arrhythmia database [31] and BUT QDB (Brno University of Technology ECG Quality Database) are used [32, 33]. To generate noisy signals, main line interference, EMG noise, and white Gaussian noise are combined with ECG signals at diverse SNRs (signal to noise ratios). The output SNR improvement (SNR), percentage root-mean-square difference (PRD), and mean square error (MSE) are used as performance metrics. To demonstrate its efficacy, the proposed denoising scheme is associated to existing techniques.

### 2.2. Empirical Mode Decomposition (EMD)

For nonlinear, multicomponent, and nonstationary time series decomposition, empirical mode decomposition is a relatively innovative signal processing technique. Since the basic purposes are straight derived from the sample signal, it differs from wavelet transform (WT) or Fourier transform (FT). The harmonics are clearly analogous to the basis function in one way or another in terms of theoretical concepts such as WT or FT. It disintegrates a signal into a quantity of oscillatory elements, which are the IMFs, according to the EMD theory (intrinsic mode functions). IMFs should share two fundamental characteristics: first, they should have the equal numeral of peaks and zero-crossings or vary by no more than one; second, they should be balanced in terms of local zero mean. Any signal's empirical mode decomposition (EMD) measures *x*(*t*) are as follows:

(1) Initially, all the limited low and high peaks of the specified signal are recognised.
(2) Three-dimensional spline exclamation is employed to link all local maxima and therefore mother signal's upper envelope is constructed.
(3) The same process is performed for the local minima to generate the inferior envelope.
(4) The mean *m*_1_ of lower and upper envelope is computed, and the alteration denoted as *f*_1_ between the signal *x*(*t*) and *m*_1_ is calculated and denoted as *f*_1_(*t*).
(5) If *f*_1_(*t*) fulfils the IMF conditions, then *f*_1_ is the first amplitude and frequency controlled oscillatory approach of *x*(*t*).
(6) In case *f*_1_ is not an IMF, then the process of shifting labelled in the steps 1 to 3 is carried out again on *f*_1_.
(7) Let us consider that after *i* operation cycles, *f*_1_*i* becomes an IMF; henceforth, it is termed as *c*1= *f*_1_*i* which is the first IMF element from the novel data.
(8) Deducting *c*1 from *x*(*t*), we get r1 which is considered as the original data for subsequent cycle.
(9) Reprocess the overhead procedure *k* epochs, and *k* number of IMFs are achieved along with the last residue *r*_*n*_. This process of decomposition can be discontinued when *r*_*n*_ turns into a monotonic function from which it is not possible to extract any more IMF. A popular criterion for stopping is to have the NSD (normalised standard difference) value inside a predetermined threshold [34] where
  (1) $$\begin{array}{c} \text{NDS}=\;\sum_{k=1}^{r}\frac{{\left|f_{i-1}\left(t\right)-f_{i}\left(t\right)\right|}^{2}}{f_{i}^{2}\left(t\right)}. \end{array}$$

### 2.3. Baseline Wander Correction

As seen in the preceding section, the EMD (empirical mode decomposition) approach disintegrates the signal into IMFs of reducing rate, and it is projected that the baseline wander is current in certain higher order IMFs. Although the EMD technique residue may encompass some complete baseline drift components, it is unlikely to contain the whole baseline problematic. This is due to the fact that the baseline wander may have several extrema and zero crosses, which are not permitted in the residue due to its properties. As a result, estimating the amount of higher order IMFs that contribute to a difference in the baseline is a challenging challenge. They should also not include any valuable information. The slope changes from fragment-to-fragment as the ECG signal is piecewise separated into smaller sections. The total number of slopes is an approximation of the sum of baseline drift. The value is equal to the baseline wander. Since low frequency IMFs include baseline segments, partial restoration of the final few IMFs including residue may mean baseline drift, but identifying the order of IMFs responsible for baseline drift is difficult. As a result, the remaining few IMFs are detached one-by-one before the global slope approaches a minimum.

### 2.4. Elimination of Power Frequency

The primary notion behind power line removal using EMD is to undertake selective reconstruction of the ECG from the IMFs, which is accomplished through the use of a computer. A high frequency component of an ECG signal is related with lower order IMFs, whereas a low frequency component is associated with higher order IMFs, as previously indicated. The fundamental theory underlying denoising via EMD is to choose a subset of IMFs that does not display noises for ECG reconstruction. It is evident that the first IMF comprises some QRS information and mostly high-frequency noise. The next few IMFs comprise helpful information pertaining to ECG as well as high-frequency noises. Also, removal of such IMFs could result in losing some key information regarding ECG, and if these are retained, the ECG information may contain some high-frequency noise.

It has been seen that on removing just the first IMF, and retaining all the others, the resulting output would include significant levels of noise, while some of the valuable high-frequency fragments would be missing. If additional IMFs are unconcerned directly, then it will distort the resulting wave at the shrill edges, particularly the *R* peak. This could be due to the sharp and high-frequency oscillation mode of the *R* peak, which is majorly represented with regards to the higher order IMFs [35]. To address this issue, a window-based QRS preservation strategy has been offered as a solution. During this procedure, the QRS area is retained until the first several IMFs are rejected, and it is then integrated with the remainder of the region once the IMF has been eliminated. The difficulty with this technique is that some noise in the QRS field is disregarded, which leads to incorrect results. For the preservation of the *R* peak during EMD-based denoising of ECG data, a model-based solution has been presented [36, 37]. However, developing a specific ECG model is difficult since the wave varies for dissimilar diseases and differs from person-to-person; it may also vary even when the person is the same due to a stressful situation or a long interval time. Furthermore, with S wave below the baseline, a sharp and long depression could be seen in some leads. The presence of a sharp and long *Q* wave in the ECG, as well as other suggestive features, can be used to diagnose such coronary artery diseases, such as myocardial infarction. In these cases, distortion of the *Q* and S peaks, as well as *R*, can occur. As a result, removing the first few IMFs for denoising has the potential to distort the entire QRS complex.

### 2.5. Data Reconstruction

Due to this, QRS complex detection can also turn erroneous. A simple algorithm has been put forward to select the required IMFs in order to deal with all of these challenges. The steps are explained as follows:

(1) First, calculation of the increasing mean pertaining to the IMFs is done. In this step, calculation of the mean of the first IMF is done. Then, one-by-one, second IMF onwards addition is done to it and in each reconstruction, calculation of mean signal is done as follows:
  (2) $$\begin{array}{c} R_{k}=\text{Mean}\left[\sum_{i=1}^{k}f\left(i\right)\right]. \end{array}$$
Since noise in a high frequency component is almost near to null mean, a zero or actual low rate of signal mean is expected to parallel with the noise. In most of the cases, noise and certain useful high-frequency component are represented by the first IMF. Thus, determination of a mean level of threshold signal is done up to which the increasing mean needs to be regarded as mean of noise signal. The set of IMFs that possess a cumulative mean that is higher than the threshold value is regarded to contain helpful information pertaining to ECG; as presented in Figure 1, mean values correspond to the first and second IMFs.
(2) To create a confirmative test, the signal strength of each IMF is measured. When power frequency noise is existing in an ECG, it is common to see small amplitude as well as high-frequency oscillation in the definite ECG suggestion. The signal power that corresponds to the noise must also be minimal due to the small amplitude. All IMFs have a moderate power band, with the exception of certain minor order IMFs (i.e., high frequency) that have a much smaller power band. It was discovered that the range of IMFs with ample lower power and those with very small signal mean values were the same. As a result, there is a possibility that these IMFs are just noise and can be missed during reconstruction.
(3) The ECG signal can be reconstructed from IMFs by adding their vectors in the following manner:
  (3) $$\begin{array}{c} \hat{ECG}=\sum_{l=1}^{r}\text{IMF}s_{l}, \end{array}$$
   where *l* is the IMFs number.

## 3. Results and Discussion

The efficacy pertaining to the put forward work has been assessed by employing the standard database mentioned in section 2.1. Time-varying QRS morphology is included in these signals, both abnormal and normal ECG beats. To the signals, addition of three virtual noises, namely, electromyogram (EMG) noise, white Gaussian noise, and main line interference at numerous SNR decibel (dB) levels ranging from 0 to 25 at 5 dB steps, is done. Then, a comparison of the put forward work's performance with those of the existing ECG denoising techniques, namely, EMD-based technique [23], NML filter [28], FIR [17], and PCA-based filter [30], is done.

Then, we performed a qualitative routine analysis for the put forward scheme via visual check.  Figure 2 shows the denoised ECG records 103 m, which has been contaminated by the white Gaussian noise at SNR level of 10 dB. As per Figure 2, a higher ability to extract the ECG data from a record with noise at minimum distortion was found associated with the ASMF-based approach. This approach also helps to preserve the processed signal's morphological properties, which include considerable clinical information.  Figure 3 demonstrates the put forward technique's denoising proficiency pertaining to an ECG signal that has been contaminated with EMG noise. Here, it was found that EMG noise at SNR level 5 dB contaminates the ECG record 100 m.  Figure 3 demonstrates that with the help of this technique, EMG noise can be efficiently removed from the signal and it also helps to retain the information.

This section describes the quantitative performance analysis pertaining to the mentioned technique. The assessment takes into account three performance metrics, namely mean square error (MSE), output signal-to-noise ratio (SNR) enhancement, and percentage root mean square difference (PRD). The study involving ECG denoising frequently employs SNR, PRD, and MSE as performance parameters [38]. SNR can be defined as the standard metric that helps to quantify a signal's quality in terms of the energy. The signal energy is defined by the SNR based on the associated noise's energy levels. SNR signifies the enhancement of SNR rate pertaining to a signal via filtering method. Because the aim of the analysis is to remove noise from the ECG signals, an increase in SNR can be considered a useful performance metric for assessing the filter's ability to reduce background noise. MSE may be used to approximate the original signal and monitor the precision of the filtering technique. During the filtering phase, it also determines the energy of the error signal. As a result, a lower MSE value indicates better estimate of the original signal as well as better signal information retention. Each portion of the ECG signal conveys a significant amount of clinical information. In medical applications, highly skewed ECGs are largely irrelevant. PRD is a performance metric that is used to assess the efficacy of various filtering strategies in relations of preserving relevant medical data during the procedure of signal extraction. Lower PRD values mean that the physiological information in highly processed ECG signals is better preserved. In this method, 100 simulations are run for each ECG record at all input SNR levels, with the mean of all results analysed appropriately. The following are the output parameters that resulted as follows:

(4) $$\begin{array}{c} \text{SNR}=10\;\log\frac{\sum_{k=1}^{N}{\left(ECG_{\text{correpted}}\left[k\right]-ECG_{\text{original}}\left[k\right]\right)}^{2}}{\sum_{k=1}^{N}{\left(\hat{\text{ECG}}\left[k\right]-ECG_{\text{original}}\left[k\right]\right)}^{2}},\\ \text{MSE}=\frac{1}{N}{\sum_{k=1}^{N}\left({\text{ECG}}_{\text{original}}\left[k\right]-\hat{\text{ECG}}\left[k\right]\right)}^{2},\\ \text{PRD}=\sqrt{\frac{\sum_{k=1}^{N}{\left({\text{ECG}}_{\text{original}}\left[k\right]-\hat{\text{ECG}}\left[k\right]\right)}^{2}}{\sum_{k=1}^{N}{\text{ECG}}_{\text{original}}^{2}\left[k\right]}}. \end{array}$$

Figure 4 shows the improved SNRs obtained for EMG noise-degraded ECG signals with input SNR levels ranging from 0 to 25 dB. Figure 4 shows that for the entire range of input SNR levels, the proposed approach outperforms the other approaches in terms of SNR. SNR decreases in proportion to increase in input SNR levels.  Figure 5 shows the output SNR levels of denoised ECG signals when Gaussian white noise is taken into account. It demonstrates that the proposed algorithm achieves a higher SNR than the other algorithms at any input SNR stage.

The mean square error (MSE) is one of the main routine schemes of measurement used to assess a denoising algorithm's effectiveness. It explains the algorithm's ability to approximate the consistency of the original signals. A lower MSE value means that the initial signal was recovered more effectively.  Figure 6 shows MSE comparisons of numerous ECG noise filtering methods in the case of EMG noise corruption. At every SNR step, it was discovered that the projected ECG denoising scheme achieves a lower MSE than other current techniques. The MSE values of the denoised ECG signals at various input SNR levels are shown in Figure 7, where the indications are degraded with Gaussian white noise at various SNR levels. It demonstrates that the proposed approach achieves a lower denoised signal MSE than other techniques. The findings point to this adaptive technique's dominance in retrieving original signals from noisy conditions.

Another parameter in quantitative analysis is the percentage root mean square difference (PRD), which measures the amount of distortion in a denoised signal. The metric defines a filtering method's ability to minimize noise without sacrificing sensitive information. The PRD value should be as low as possible for reduced distortion and superior recapture of the initial data.  Figure 8 shows a PRD value assessment of signal recovery in the case of EMG noise corruption. The proposed approach achieves lower PRD values across all input SNR levels, implying that it is more capable of minimizing EMG noise in ECG signals.  Figure 9 shows a performance comparison of the PRD values for Gaussian white noise. The proposed approach yields lower PRD values at all input SNR levels, implying that clinical information is better preserved in filtered signals with lower distortion.

In the automated processing of ECG signals, noise reduction is still important. The aim of this study is to combine the benefits of EMD and adaptive process to eliminate noise in ECG signals while reducing distortion. EMD processes use their data-driven versatility to efficiently decompose signals into IMFs as the oscillation changes. Finally, combining the suggested technique with the ideal restoration process results in superior recovery of initial ECG signals with less alteration. For a simulation study, three forms of noise are inserted into the original ECG recordings, each with a different SNR level.

Figures 2 and 3 both describe qualitative investigation of the recovered data signals across various noise cases. Closer observation of the abovementioned figures show that recovered signal quality using the proposed approach is superior to other schemes. Processed signals are shown to contain detailed local features that appropriately express abundant clinical information. In quantitative analysis, the 3-performance metrics of SNR, PRD, and MSE are used. Figures 4 and 5 both show that the proposed method attains larger SNRs for denoised signal quality in comparison to the other current methods, with consideration of powerline interference and Gaussian noise. Figures 6 and 7 both represent the usefulness of the suggested method with regards to MSE. At every input SNR level in the range 0 dB−25 dB, the MSE attained by the proposed method is lower than that of the other techniques, which suggests that this approach estimates the initial ECG signal with a lower error. PRD value indicates the quality of processed signals with regards to clinical use. Figures 8 and 9 both show that this approach results in a lower PRD rate than that of the other approaches used for resolving EMG interference and Gaussian noise.

## 4. Conclusion

In this study, an adaptive ECG denoising process derived from EMD is proposed. The core objective of this research is to improve on the conventional strategy of relying on EMD for ECG denoising, through adaptive calculation of lower IMF mean values in the reconstruction of original signals. In classic EMD-based ECG noise removal approaches, cancellation of initial IMFs using a window-based method is applied in order to reduce high-frequency noise. Nevertheless, these strategies tend to degrade either high-frequency detail in ECG signals or else ignore noise in the QRS complex region. Classic EMD-based methods differ in the fact that a mean calculation is used to reject high-frequency noise while preserving QRS complexes. The standardised MIT-BIH and Brno University of Technology ECG Quality Database (BUT QDB) and ECG signal databases are used in the simulation analysis. A general noise, specifically Gaussian white noise in combination with EMG noise, is added to test signals at different input SNR levels. The 3 parameters for performance evaluation SNR, PRD, and MSE are used to evaluate the efficiency of the proposed approach. The efficiency of this technique is then compared with that of the NML filter [28], EMD-based [23], FIR [17], and PCA-based filter [30] ECG noise removal strategies. It was noted from simulation studies and detailed investigation that the proposed ECG noise filtering technique outperforms the current methods. A thorough inspection of the resulting performances suggests that the proposed scheme can be standardised as a tool for reducing noise in ECG signals pathology. This approach will be useful for developing computerised computational interpretation systems in the future.

## Figures and Tables

**Figure 1:** The proposed method.

**Figure 2:** The denoising of ECG signal.

**Figure 3:** Noisy and clean signal.

**Figure 4:** The improved SNRs obtained for EMG noise-degraded ECG signals.

**Figure 5:** The output SNR levels of denoised ECG signals (Gaussian noise effect).

**Figure 6:** The MSE comparisons of numerous ECG denoising methods in the case of EMG noise.

**Figure 7:** The MSE values of the ECG signals noise filtering at various input SNR levels.

**Figure 8:** The PRD value evaluation of signal recovery in the case of EMG noise corruption.

**Figure 9:** The routine comparison of the PRD values for Gaussian white noise.

## Data Availability

The data used to support the findings of this study were obtained from the MIT-BIH arrhythmia database and the BUT QDB (Brno University of Technology) database.
